RETRACTED

# Efficacy and Mechanism of Roxadustat plus Oral Iron in the Treatment of Elderly Chronic Kidney Disease with Anemia

**DOI:** 10.1155/2022/9192655

**Published:** 2022-06-25

**Authors:** Bo Liu, Tiantian Shi, Shaojiang Tian, Xianrui Luo, Chen Yang, Jing Wen

**Affiliations:** ^1^Department of Nephrology, Renmin Hospital, Hubei University of Medicine, Shiyan, Hubei, China; ^2^Department of Blood Purification Center, Renmin Hospital, Hubei University of Medicine, Shiyan, Hubei, China

## Abstract

**Objective:**

For investigating the efficacy and mechanism of Roxadustat + oral iron in the treatment of elderly chronic kidney disease (CKD) complicated with anemia.

**Methods:**

A total of 100 elderly patients with CKD and anemia admitted to our hospital between April 2020 and December 2021 were enrolled as research subjects, and the patients were assigned to control group (Con group, *n* = 50) or experimental group (Exp group, *n* = 50). The patients in the Con group were given oral iron, and those in the Exp group were given Roxadustat capsule based on the Con group. Both groups were given subcutaneous injection of recombinant human erythropoietin. The clinical efficacy, anemia indexes, iron metabolism indexes, inflammatory indexes, and adverse reactions were compared between the two groups.

**Results:**

The Exp group showed a notably higher treatment effective rate than the Con group (*P* < 0.05). After treatment, the anemia indexes, iron metabolism indexes, and inflammatory indexes in the Exp group were notably better than those in the Con group (*P* < 0.05). The Exp group showed a notably lower incidence of adverse reactions during treatment than the Con group (*P* < 0.05).

**Conclusion:**

Roxadustat plus oral iron yields a pronounced clinical efficacy in the therapy of elderly patients with CKD and anemia.

## 1. Introduction

Chronic kidney disease is a chronic structural and functional disease of the kidneys caused by damaged renal blood vessels, renal tubules, and other diseases such as glomerulonephritis [1]. There are 5 clinical stages of chronic kidney disease (CKD), of which the third stage is the turning point of the disease. Patients in the third stage experience symptoms such as edema, hematuria, and proteinuria, leading to renal dysfunction, end-stage renal failure, and even various complications such as cardiovascular diseases [2]. Anemia, one of the main clinical manifestations of patients with CKD, occurs in the early stage of the patient's disease and results in weak renal function, raising the complexity of the therapy of patients with CKD, and increasing the mortality rate [3]. Clinical studies have shown that the relative or absolute insufficiency of erythropoietin caused by renal damage and the insufficiency of basic raw materials required for the synthesis of hemoglobin are the main factors leading to CKD with anemia [4]. Recombinant human erythropoietin is a drug recommended universally for the therapy of CKD with anemia. Despite the reduction of blood transfusion by increasing the patient's hemoglobin level, the patient is vulnerable to autoinflammation and iron deficiency, which abates the effectiveness of recombinant human erythropoietin in the therapy of patients with CKD and anemia [5]. Therefore, iron supplementation is of much concern for elderly patients with CKD and anemia. However, researchers [6] pointed out that patients are prone to acute and chronic iron toxicity under the impact of overdose free iron [7, 8]. Also, anemia is associated with low immune function, myocardial damage, and hypoxia. Modern medicine believes that the decreased secretion of erythropoietin (EPO) produced by the kidneys, insufficient raw materials such as iron and folic acid and the inhibition of bone marrow hematopoiesis are contributors to CKD with anemia [9, 10]. EPO is an active glycoprotein secreted by the kidney, which stimulates erythrocyte proliferation through binding to EPO receptors on the surface of erythrocytes. Evidence supported that EPO can substantially improve the clinical indicators of patients with CKD and anemia [11]. Clinically, symptomatic therapy and iron supplements are used to treat CKD with anemia, that is, subcutaneous injection of recombinant human erythropoietin, supplemented by iron [12]. However, some patients are prone to headache, epilepsy and other symptoms, as well as allergic reactions and blood hypercoagulability after therapy with recombinant human erythropoietin [13]. Oral iron is associated with adverse reactions such as gastrointestinal irritation. Roxadustat is a hypoxia-inducible factor prolyl hydroxylase inhibitor developed in recent years that can correct anemia via multiple pathways by inactivating prolyl hydroxylase Enzyme (PHD) under hypoxia, and regulating the main transcription factor of EPO gene; under normal circumstances, HIF-*α* and HIF-*β* that can be hydroxylated by PHD and degraded by the body bind to the nucleus and further bind to the hypoxia response element, thereby mediating gene transcription [14]. Hypoxia-inducible factor prolyl hydroxylase inhibitor induces functional HIF transcriptional response by stabilizing HIF and inhibiting PHD, and promotes the expression of erythropoietin receptor while promoting the production of endogenous EPO, thereby improving anemia. HIF-PHI inhibits hepcidin expression and increases Hb level, which is a favorable therapy approach for patients who do not receive hemodialysis. Roxadustat is the only new drug on the market for HIF-PHI, which can improve the absorption, utilization, and transport of iron, and comprehensively regulate the production of red blood cells. Our hospital also believes that traditional Chinese medicine is practical to treat elderly patients with CKD and anemia. Accordingly, this study was performed for exploring the efficacy of the Roxadustat + oral iron + traditional Chinese medicine in the therapy of elderly CKD with anemia.

RETRACTED

## 2. Materials and Methods

### 2.1. Patients Profile

A total of 100 elderly patients with CKD and anemia treated in our hospital between April 2020 and December 2021 were enrolled as the research subjects, and the patients were assigned to the control group (Con group, *n* = 50) or the experimental group (Exp group, *n* = 50) in the light of different therapy methods. The Con group was composed of 27 males and 23 females at 61–78 years old (average age: (65.42 ± 4.28) years); CKD stages: 28 cases of stage 3, 17 cases of stage 4, and 5 cases of stage 5. The Exp group was composed of 28 males and 22 females, at 61–79 years old (average age: (65.45 ± 4.32) years); CKD stages: 26 cases of stage 3, 19 cases of stage 4, and5 cases of stage 5. The baseline data in the two groups were balanced (Table 1). The studies involving human participants were reviewed and approved by the Renmin Hospital, Hubei University of Medicine, No.10773/71.

### 2.2. Inclusion and Exclusion Criteria

#### 2.2.1. Inclusion Criteria

Inclusion criteria were defined as follows: (1) the patients who met the clinical diagnostic criteria for CKD; (2) aged >60 years; (3) the patients who met the clinical diagnostic criteria for anemia (male: 60 g/L ≤ Hb < 130 g/L; female: 60 g/L ≤ Hb < 120 g/L); and (4) the patients and their families who provided signed informed consent forms.

#### 2.2.2. Exclusion Criteria

Exclusion criteria were defined as follows: (1) patients with CKD on dialysis; (2) patients with active bleeding; (3) patients with malignant tumors; (4) patients with blood transfusion history 1 month before enrollment were excluded (5) patients with malnutrition; (6) patients with severe organ failure such as liver and kidney; and (7) patients with mental disorders.

### 2.3. Methods

Both groups of patients were given high-quality low-protein diet, blood pressure, water, electrolyte and acid-base balance adjustment and other conventional treatments. At the same time, both groups were given subcutaneous injection of recombinant human erythropoietin injection (CHO cells) (specification: 1 ml: 3000 IU), 75–100 IU/kg a week, 2-3 times a week; When the hemoglobin level improves, adjust the injection dose in time to keep the patient's hemoglobin level within the range of 100–120 g/L. On this basis, the Con group was given oral iron polysaccharide iron compound capsules (specification: 0.15 g), 0.15 g once, twice a day, on an empty stomach; the Exp group was additionally given Roxadustat capsules orally (specification: 50 mg), 70 mg (for those with a body weight of 40–59 kg) or 100 mg (for those with a body weight of ≥60 kg), 3 times a week. The two groups were given 3 consecutive months of treatment.

RETRACTED

At the same time, traditional Chinese medicine treatment was given as a support treatment. Yishen Xiezhuo Recipe (Astragalus, *Lycium barbarum*, Danshen, Motherwort, Rhubarb, Alisma, and Gangmei Powder) was given 1 packet each time, orally 3 times a day.

### 2.4. Outcomes

(1) Clinical efficacy: referring to the “Guidelines for Clinical Research on New Chinese Medicines: Trial Implementation” [8], the clinical efficacy of elderly patients with CKD and anemia was evaluated according to the improvement of clinical symptoms and the increase of Hb and Hct after therapy. Markedly effective: the patients' clinical symptoms are significantly mitigated, and the increase in Hb is greater than 20 g/L and/or Hct is greater than 10%; effective: the patients' clinical symptoms are mitigated, and the increase in Hb is greater than 10 g/L and (or) Het increased by >5%; ineffective: the patient's clinical symptoms remain unchanged, and Hb and Het did not change. Total effective rate = (markedly effective + effective) number of cases/the sum of cases × 100%. (2) Anemia indicators: the fasting cubital venous blood in the morning before and after therapy was collected, and the levels of anemia indicators such as red blood cell count (RBC), hematocrit (Ha), as well as hemoglobin (Hb) were measured by a blood cell analyzer. (3) Iron metabolism indicators: the fasting cubital venous blood was acquired in the morning before and after therapy, and the patient's transferrin (TRF), ferritin (Fer), serum iron (Fe), total iron binding capacity (TIBC), and other indicators of iron metabolism were quantified via an automatic biochemical analyzer. (4) Inflammatory indicators: enzyme-linked immunosorbent assay was adopted for determining the levels of inflammatory indicators such as C-reactive protein (CRP) and interleukin 6 (IL-6), as well as interleukin 8 (IL-8) before and after therapy. (5) Adverse reactions: the adverse reactions including nausea, vomiting, diarrhea, allergy, and thrombosis were recorded by medical staff in our hospital.

### 2.5. Statistical Processing

All data analysis was conducted via SPSS 21.0 software. Measurement data (*x* ± *s*) were compared via the independent samples *t* test; count data are presented by number of cases (rate) and compared via the chi-square test. *P* < 0.05 denotes a notable difference. GraphPad Prism 8 was used for graphics rendering.

RETRACTED

## 3. Results

### 3.1. Clinical Efficacy

The Exp group showed a notably higher effective therapy rate than the Con group (*P* < 0.05, Table 2).

### 3.2. Anemia Indicators

Before therapy, the two groups were similar in anemia index (*P* > 0.05); after therapy, the Exp group showed notably better anemia index than the Con group (*P* < 0.05, Figure 1).

### 3.3. Iron Metabolism Indicators

Before therapy, the two groups were similar in iron metabolism indexes (*P* > 0.05); after therapy, the Exp group showed notably better iron metabolism indexes than the Con group (*P* < 0.05, Figure 2).

### 3.4. Inflammatory Indicators

Before therapy, the two groups were similar in inflammatory indexes (*P* > 0.05); after therapy, the Exp group showed notably better inflammatory indexes than the Con group (*P* < 0.05, Figure 3).

### 3.5. Adverse Reactions

The Exp group showed a notably lower incidence of adverse reactions during therapy than the Con group (*P* < 0.05, Table 3).

## 4. Discussion

Clinically, anemia is characterized by reduced volume of human peripheral red blood cells [8], and is associated with weakened immune function, and in severe cases, it myocardial dysfunction and lack of oxygen in severe cases [9, 10]. EPO is an active glycoprotein secreted by the human kidney, which can stimulate the proliferation of red blood cells through binding to EPO receptors on the surface of red blood cells. Clinical research has confirmed that EPO can substantially improve the clinical indicators of patients with CKD and anemia. At present, drugs such as recombinant human erythropoietin and oral iron are often used clinically to treat CKD with anemia. However, some patients are susceptible to headaches and epilepsy after therapy with recombinant human erythropoietin, and even allergic reaction, hypercoagulable state [11, 12].

HIF-PHI induces the transcriptional response of functional HIF in patients by stabilizing HIF and inhibiting PHD. It not only promotes the production of endogenous EPO in the body, but also promotes the expression of erythropoietin receptors in the body, thereby improving the patient's health [13]. Moreover, HIF-PHI inhibits the expression of hepcidin in the patient's body, thereby increasing the level of Hb. Roxadustat is the only new drug on the market for HIF-PHI, which can effectively improve the absorption, utilization and transport of iron in patients, and help patients regulate the production of red blood cells.

RETRACTED

In this study, we found that Roxadustat + oral iron resulted in higher clinical efficacy and better anemia indexes and metabolism indexes. These findings suggest that Roxadustat plus oral iron contributes to mitigate the anemia symptoms in elderly patients with CKD and anemia, and facilitate the metabolism. The results may attributed to the fact that Roxadustat can reduce the hepcidin of the patient's body, thereby increasing the TRF level of the patient's body and helping the patient to stabilize the body's Fe level [14, 15]. Rubeor et al. revealed that the level of inflammatory factors in patients with CKD and anemia may have a certain relationship with the disease, and over half of the patients are accompanied by active inflammatory response [16, 17]. de Lecea have found that inflammatory factors can increase the level of hepcidin in the patient's body, thereby inhibiting the production of EPO in the patient's kidneys, and aggravating the anemia [18]. In this study, we observed that Roxadustat + oral iron led to a milder inflammatory response. Presumably, Roxadustat alleviates the level of inflammatory indicators in the patient's body by promoting the erythropoietin receptor expression in the patient's body [19]. In terms of therapy safety, Zhang et al. [20] pointed out that high-dose recombinant human erythropoietin injection will affect the blood pressure of patients with CKD, with low but stable EPO level produced by HIF-PHI. In this study, we noted that Roxadustat + oral iron was associated with fewer adverse reactions, indicating that Roxadustat + oral iron may have a good safety profile. The possible explanation is that HIF-PHI can effectively promote the production of endogenous EPO in patients, thereby accelerating the production of red blood cells in patients, and mitigating the symptoms of anemia in patients [21–23]. In traditional Chinese medicine, the etiology and pathogenesis of renal anemia in CKD is mainly “kidney deficiency with damp-heat and blood stasis,” and the lesions are mainly located in the spleen, kidney and liver. Clinical research on anemia confirmed that the combination of “Yi Shen method” and “Xiezhuo method” is of great significance for the therapy of renal anemia, especially in patients with mild to moderate anemia. Similarly our findings are in consistent with the above-mentioned.

## 5. Conclusion

The clinical efficacy of Roxadustat plus oral iron in the therapy of elderly patients with CKD and anemia is pronounced. It improves the anemia index of patients, regulates iron metabolism, lessens inflammatory response conditions, and reduces the occurrence of adverse reactions during therapy. However, this study was conducted on elderly patients with CKD, and the robustness and generalizability of the findings are moderated by the restricted sample population. Further clinical trials are, however, required prior to general use in clinical practice.

RETRACTED

## Figures and Tables

**Figure 1:** Comparison of anemia indicators between the two groups of patients (*x* ± *s*). Note: ^*∗*^means *P* < 0.05. Before treatment, the Hb of the control group was (91.28 ± 8.25) g/L, the RBC was (2.02 ± 0.52) × 10^12^/L, the Hct was (20.73 ± 3.15)%, and the Hb of the experimental group was (91.14 ± 8.36) g/L, the RBC was (2.04 ± 0.49) × 10^12^/L, the Hct was (20.72 ± 3.21)%, and the difference was not statistically significant (*t* = 1.325, 1.247, 2.364; *P*=0.214, 0.365, 0.457). After treatment, the Hb of the control group was (121.34 ± 11.59) g/L, the RBC was (2.87 ± 0.65) × 10^12^/L, the Hct was (30.11 ± 4.12)% and the Hb of the experimental group was (132.53 ± 11.47) g/L, RBC was (3.53 ± 0.62) × 10^12^/L, the Hct was (36.37 ± 4.18)%, and the difference was statistically significant (*t* = 2.645, 4.365, 3.644; all *P* < 0.05).

**Figure 2:** Comparison of iron metabolism indexes between the two groups of patients (*x* ± *s*). *Note*: ^*∗*^means *P* < 0.05. Before treatment, the TRF of the control group was (1.71 ± 0.54) g/L, Fer was (274.10 ± 11.31) ng/ml, Fe was (10.12 ± 3.03) *μ*mol/L, TIBC was (41.83 ± 3.32) *μ*mol/L; the TRF of the experimental group was (1.73 ± 0.51) mg/L, Fer was (273.58 ± 12.02) ng/L, Fe was (10.08 ± 3.10) *μ*mol/L, and TIBC was (42.09 ± 3.17) *μ*mol/L, and the differences were not statistically significant (*t* = 3.364, 1.453, 4.647, 3.124; *P*=0.364, 0.415, 0.563, 0.524). After treatment, TRF of the control group was (2.25 ± 0.25) g/L, Fer was (185.34 ± 5.67) ng/ml, Fe was (16.23 ± 4.12) *μ*mol/L, TIBC was (49.21 ± 4.22); TRF of experimental group was (3.03 ± 0.43) g/L, Fer was (170.22 ± 5.08) ng/L, Fe was (23.21 ± 3.77) *μ*mol/L, TIBC was (56.28 ± 5.34) *μ*mol/L, and the differences were statistically significant (*t* = 2.647, 2.344, 3.154, 4.444; all *P* < 0.05).

**Figure 3:** Comparison of inflammatory indicators between the two groups of patients (*x* ± *s*). *Note*: ^*∗*^means *P* < 0.05. Before treatment, CRP of the control group was (12.13 ± 2.32) mg/L, IL-6 was (83.60 ± 9.21) ng/L, IL-8 was (81.99 ± 12.12) ng/L; CRP of the experimental group was (12.24 ± 2.30) mg/L, IL-6 was (83.78 ± 8.89) ng/L, IL-8 was (82.10 ± 12.05) ng/L, and the differences were not statistically significant (*t* = 2.354, 1.033, 3.634; *P*=0.364, 0.415, 0.524). After treatment, the CRP of the control group was (10.20 ± 1.13) mg/L, the IL-6 was (71.14 ± 6.28) ng/L, the IL-8 was (61.23 ± 3.58) ng/L; the CRP of the experimental group was (6.15 ± 0.35) mg/L, IL-6 was (42.22 ± 5.16) ng/L, IL-8 was (30.94 ± 4.58) ng/L, and the differences were statistically significant (*t* = 3.640, 3.574, 4.364; all *P* < 0.05).

RETRACTED

**Table 1:** Patients profile.

	Control group (*n* = 50)	Experimental group (*n* = 50)	*T*/*x*^2^	*P*
Gender			0.04	0.841
Male	27	28		
Female	23	22		

Mean age (years, *x* ± *s*)	65.42 ± 4.28	65.45 ± 4.32	−0.035	0.972

Chronic kidney disease staging			0.185	0.667
Stage 3	28	26		
Stage 4	17	19		
Stage 5	5	5		

**Table 2:** Clinical efficacy (*n* (%)).

	Control group (*n* = 50)	Experimental group (*n* = 50)	*x* ^2^	*P*
Markedly effective	24 (48.0)	38 (76.0)		
Effective	15 (30.0)	11 (22.0)		
Ineffective	11 (22.0)	1 (2.0)		
Total (%)	39 (78.0)	49 (98.0)	9.47	0.002

**Table 3:** Adverse reaction (*n* (%)).

	Control group (*n* = 50)	Experimental group (*n* = 50)	*x* ^2^	*P*
Nausea and vomiting	4 (8.0)	1 (2.0)		
Diarrhea	2 (4.0)	0 (0)		
Allergies	1 (2.0)	1 (2.0)		
Thrombus	3 (6.0)	0 (0)		
Total	10 (20.0)	2 (4.0)	6.061	0.014

## Data Availability

All data generated or analysed during this study are included in this published article.
